The article "Analgesic Effects of Epidural Labor Analgesia at Different Periods and Its Effects on Maternal and Infant Outcomes and MiRNA-146b Level" was published in 2021. Journal: J Healthc Eng.

# Analgesic Effects of Epidural Labor Analgesia at Different Periods and Its Effects on Maternal and Infant Outcomes and MiRNA-146b Level

**DOI:** 10.1155/2021/2879678

**Published:** 2021-11-25

**Authors:** Lihong Wang, Hui Liu, Ye Duan, Qingyu Cheng, Suhua Feng

**Affiliations:** ^1^Department of Anesthesiology, Chifeng Obstetrics and Gynecology Hospital, Chifeng 024000, Inner Mongolia, China; ^2^Department of Anesthesiology, The Affiliated Hospital of Inner Mongolia Medical University, Hohhot 010010, Inner Mongolia, China

## Abstract

This paper aimed to analyze the analgesic effects of continuous epidural labor analgesia (ELA) at different periods and its effects on postpartum depression, maternal and infant outcomes, and maternal blood pressure. Giving birth in our hospital from September 2017 to August 2019, 119 primiparas with spontaneous delivery were enrolled and divided into an observation group (65 cases) and a control group (54 cases). Patients in the observation group received epidural block analgesia in advance, whereas those in the control group received epidural block analgesia routinely. At 25 days after delivery, breast milk samples were collected, in which miRNA-146b level was detected by PCR. The patients were compared between the two groups with respect to progress of labor, analgesic effects during 3 stages of labor, labor outcomes, adverse reactions, and levels of NO, ANP, and ET-1 in the parturients' umbilical artery blood. Compared with those in the control group, patients in the observation group had a remarkably higher miRNA-146b level in the breast milk (*P* < 0.05), remarkably lower average Visual Analogue Scale (VAS) scores during the active phase and the second stage of labor (*P* < 0.05), and remarkably higher levels of NO, ANP, and ET-1 (*P* < 0.05). There were no statistically significant differences in adverse reactions and modes of delivery between the two groups (*P* < 0.05). ELA starting from the latent phase can improve the miRNA-146b level in maternal breast milk, alleviate labor pain of parturients, and shorten stages of labor. Therefore, our study is worthy of clinical promotion. We still need to do more experiments and use more data to conclude more scientific results in future research work.

## 1. Introduction

During delivery, parturients experience uterine contraction (UC) induced pain, which causes hemodynamic changes (such as increases in heart rate and blood pressure) and negative emotions (such as anxiety). With the development of medicine, it is generally believed that childbirth without pain (CWP) is helpful to improve the feeling of childbirth and pregnancy outcomes [1,2], so the way to relieve parturients' pain during delivery and prevent it has been become an important evaluation indicator for measuring delivery quality also a research direction of modern obstetrics [3,4].

Patient-controlled epidural analgesia (PCEA) is widely used during delivery due to its good analgesic effect and mild motor block, with its application in developed countries of 61%–75% [5]. Previous views held that the late latent phase or early active phase (3-4 cm of the cervix) of stages of labor is a relatively suitable time for labor analgesia, which is rarely used in the early latent phase, but this view has not been clearly verified because the stimulation of pain in the latent phase brings adverse effects on mothers and infants [6,7]. MicroRNAs (miRNAs) are a kind of small RNAs of endogenous noncoding proteins, composed of 20–25 nucleotides [8]. They are recently found expressed in human milk and other body fluids, with immune-related miR-146b particularly expressed [9]. MiRNAs in human milk can tolerate the acid environment and enzymolysis of the gastrointestinal tract, suggesting that they may be directly absorbed by infants and involved in their immune regulation [8]. The component of human milk is affected by maternal factors (such as mother's age, nutritional status, pregnancy complications, and modes of delivery) and infant factors [10,11]. Therefore, we observed immune-related miR-146b expression in human milk for epidural labor analgesia (ELA) at different periods in this study.

For exploring the influences of ELA at different periods on labor outcomes, 119 primiparas admitted to our hospital were enrolled as the research objects in this study. The clinical application effects of ELA at different times and its influences on the occurrence of adverse reactions and miR-146b expression were investigated to provide reference for clinical application.

## 2. Materials and Methods

### 2.1. General Information

A total of 119 primiparas admitted to our hospital from September 2017 to August 2019 were enrolled as the research objects. They were aged 20–32 years. Their average age was 27.58 ± 4.57 years, their gestational week was 37–42 weeks, and their average gestational week was 39.78 ± 0.85 weeks. All primiparas did not have pregnancy complications during the whole pregnancy, and those with the taboo of breastfeeding were excluded. All primiparas were divided into the observation group (those aged 26.83 ± 3.81 years with a gestational week of 36.62 ± 1.42 weeks) and the control group (those aged 27.49 ± 3.11 years with a gestational week of 36.39 ± 1.66 weeks) based on the period of ELA. Inclusion criteria: those with single head position; those with no contraindication to epidural anesthesia; those with a gestational week >37 weeks; those requiring labor analgesia; and those with the ASA classification of grades I-II. Exclusion criteria: those with breech or transverse position; those with pregnancy complications; those with coagulation disorders or blood platelet disorders; those complicated with abnormal complications (such as premature rupture of membranes, fetal distress, and cephalopelvic disproportion), cord around the neck for >2 weeks, and estimated fetal weight >3500 g; and those with a high-risk pregnancy.

### 2.2. Methods

ELA was conducted when the cervix was opened 1 cm for primiparas in the observation group and 2-3 cm for those in the control group. L2-3 space was selected as the puncture point, with an epidural catheter inserted towards the direction of the head for approximately 4 cm depth. Firstly, 1% lidocaine (3–5 mL) was injected, and then 10 mL of mixed solution (0.1% ropivacaine and 0.5 *μ*g/mL sufentanil) was given if there was no blood vessel insertion or spinal anesthesia, and a patient-controlled analgesic pump was finally connected if there were no adverse reactions. The loading dose was 10 mL. The background dose was 5 mL/h, the single dose was 5 mL, and the locking time was 15 min. Labor analgesia was stopped when the cervix was fully opened. During labor analgesia, electrocardiograms and blood oxygen saturation were closely monitored. If blood pressure dropped by 20% compared with that before analgesia, compound sodium chloride should be intravenously dripped rapidly. If the blood pressure dropped by more than 30%, 6 mg of ephedrine should be given. If blood oxygen saturation was lower than 95%, appropriate oxygen inhalation should be given. During operation, obstetric management was determined by obstetricians and midwives according to the fetus, UC progression, etc.

### 2.3. qRT-PCR for MiR-146b Level in Breast Milk

At 25 days after delivery, breast milk samples were collected, in which the miRNA-146b level was detected by PCR. The samples were taken out of the refrigerator, melted on ice, and centrifuged twice (1200 × *g*, 4°C, 10 min). The degreased supernatant was centrifuged again (21500 × *g*, 4°C, 60 min) to remove the remaining fat, protein, and cell debris. The supernatant obtained passed through a polyvinylidene fluoride (PVDF) membrane with a diameter of 0.45 *μ*m, and the residual cell debris was removed to obtain whey. miRNeasyMiniKit (Qiagen, Germany) was used to extract total RNA from the whey. The extracted RNA was dissolved to 25 *μ*L with diethyl pyrophosphate (DEPC), and its concentration and purity were detected by an UV spectrophotometer. It was reversely transcribed by poly(A) tailed RT-PCR. The specific process was as follows: gRNA (2 *μ*g) was added into a 20 *μ*L reverse transcription system for reaction at 37°C for 60 min, and the 3′-end of miRNAs was poly(A) tailed; next, a certain amount of poly(A) modified miRNAs was taken for reaction at 37°C for 60 min, so as to conduct a reverse transcription reaction. After the reverse transcription product cDNA was diluted 10 times, U6 was used as the internal reference for fluorescence quantitative PCR (qRT-PCR) to detect the miR-146b level in the breast milk. qRT-PCR was performed to detect the level with the external reference used as a control. The conditions were 94°C for 2 min, 94°C for 20 s, and 60°C for 34 s, for a total of 40 cycles. After the reaction, melting curves were analyzed immediately to determine whether nonspecific amplification existed. The miR-146b level in the breast milk was calculated by 2^−ΔΔCt^, during which 3 same wells were set in each group. Forward and reverse primer sequences of miR-146b were 5′-CGGCACTGAGAACTGAATCC-3′ and 5′-CAGTGCAGGGTCCGAGGTATC-3′. Those of U6 were 5′-TGCGGGTGCTCGCTCGGCAGC-3 and 5′-GTGCAGGGTCCGAGGT-3′.

### 2.4. Observational Indicators

Modes of delivery and levels of NO, ANP, and ET-1 in the parturients' umbilical artery blood were compared between the two groups. The Visual Analogue Scale (VAS) [12] was used to score pain. Zero is painless. A score of 1–3 points is slight pain that patients can tolerate. A score of 4–6 points is tolerable pain that affects sleep. A score of 7–10 points is intolerable pain. VAS scores were recorded every 15 min. The parturients' average VAS scores of different stages of labor (latent phase, active phase, the second stage of labor, and the third stage of labor) were recorded. The parturients' adverse reactions were compared between the two groups, including respiratory depression, nausea and vomiting, and numbness of limbs. At 25 days after delivery, breast milk samples were collected, in which the miRNA-146b level was detected by PCR.

### 2.5. Statistical Analysis

The data generated in this experiment were analyzed and processed by SPSS v22.0. Measurement data were expressed by mean ± standard deviation ($\bar{x}$ ± *s*), and their comparison between groups was analyzed by *t*-test. Count data were analyzed by *X*^2^ test. When *P* < 0.05, the difference was statistically significant.

## 3. Results

### 3.1. Comparison of General Information

There were no statistically significant differences between the observation and control groups in terms of general information such as age, gestational week, body mass index (BMI), types of parturients, and blood pressure (*P* > 0.05), which indicated comparability (see Table 1).

### 3.2. Comparison of Labor Duration

Labor duration in the observation and control groups was recorded. According to the *t*-test, the latent phase in the first stage of labor was longer in the control group, with no statistically significant differences in the active phase in the first stage of labor, in the second stage of labor, and in the third stage of labor between the two groups (*P* > 0.05) (see Table 2).

### 3.3. Comparison of Modes of Delivery

Parturients in the observation and control groups had no forceps delivery. There were no statistically significant differences between the two groups in cesarean section and spontaneous delivery rates (*P* > 0.05) (see Table 3).

### 3.4. Comparison of NO, ANP, and ET-1 Levels

Levels of NO, ANP, and ET-1 in the parturients' umbilical artery blood were remarkably higher in the observation group than those in the control group (*P* < 0.01) (see Table 4 and Figure 1).

Comparison of NO level in the parturients' umbilical artery blood between the observation and control groups (A): the level was remarkably higher in the observation group. Comparison of ANP level in the parturients' umbilical artery blood between the observation and control groups (B): the level was remarkably higher in the observation group. Comparison of ET-1 level in the parturients' umbilical artery blood between the observation and control groups (C): the level was remarkably higher in the observation group.

### 3.5. Comparison of VAS Scores at Different Time Points

VAS scores were not statistically and significantly different between the observation and control groups at the latent phase and the third stage of labor (*P* > 0.50). The average VAS scores at the active phase and the second stage of labor were remarkably lower in the observation group (*P* < 0.05) (see Table 5 and Figure 2).

Comparison of VAS score at the latent phase in the first stage of labor between the observation and control groups (A): the score was not statistically and significantly different between the two groups. Comparison of VAS score at the active phase in the first stage of labor between the observation and control groups (B): the score was remarkably lower in the observation group. Comparison of VAS score at the second stage of labor between the observation and control groups (C): the score was remarkably lower in the observation group. Comparison of VAS score at the third stage of labor between the observation and control groups (D): the score was not statistically and significantly different between the two groups.

### 3.6. Comparison of Adverse Reactions

Neither the observation group nor the control group had respiratory depression. There were 12 cases (18.46%) of nausea and vomiting in the observation group and 3 cases (5.56%) in the control group, with a significant difference (*P* < 0.05). There were 2 cases (3.08%) of numbness of limbs in the observation group and 3 cases (5.56%) of numbness of limbs in the control group, with no significant difference (*P* > 0.05) (see Table 6).

### 3.7. Comparison of MiRNA-146b Level

The miRNA-146b level in the breast milk was remarkably higher in the observation group than that in the control group (*P* < 0.05) (see Table 7).

The level of mir-146b in the observation group was significantly higher than that in the control group.

## 4. Discussion

Pain during delivery is a severe stress reaction. UC, cervical dilatation, and vaginal vulvar traction in late delivery are introduced through splanchnic and perineal nerves, resulting in the increased secretion of hormones such as endorphin, catecholamine, and epinephrine in maternal blood, elevated blood pressure, and aggravated cardiac load [13,14]. At the same time, electrolyte disturbances caused by tachypnea in parturients are easy to cause their and fetuses' hypoxemia, as well as fetal distress [15]. Delivery pain also leads to UC, uncoordinated cervical dilatation, prolonged stage of labor, and a series of adverse reactions [16]. The longer the stage of labor is, the deeper the adverse effects are. ELA in an appropriate timing can relieve primiparas' pain and shorten their stage of labor, so the appropriate timing of labor analgesia is clinically significant [17].

Having become the standard scheme for labor analgesia, epidural block labor analgesia can block pain stimulation, reduce the secretion of neurotransmitters, and eliminate influences of maternal mental factors on force and stage of labor, as well as make UC regular, accelerate cervical dilatation, and have less motor block [18–20]. In this study, analgesia was performed on the delivered parturients at latent and active phases. The average VAS scores at the active phase and the second stage of labor were remarkably lower in the observation group than those in the control group, which shows that the analgesic effect is remarkably better in the observation group. The latent phase was shorter in the observation group, with no statistically significant differences in the second and third stages of labor between the two groups, indicating that ELA at the latent phase is effective in shortening the stage of labor. Hormones and autocrine-paracrine regulatory mechanisms in mothers can affect umbilical cord angiogenesis and thus play a role in regulating blood flow. Vascular endothelial cells have two regulatory substances, vasodilator, and vasoexcitor materials. NO and ANP are the main vasodilator materials, while ET is the main vasoexcitor material. The three can dilate and contract vascular smooth muscles to regulate blood supply [21, 22], also existing in the umbilical vascular endothelium. ET-I belonging to ET can enhance ANP and NO expression, and ANP has natriuretic, diuretic, and vasodilative effects. When blood volume increases, ET-1 secretion can be stimulated to increase first and then affect ANP and NO, playing a vasodilative role [23, 24]. ELA blocks sympathetic nerves, relieves pain-induced spasms on small vessels, and improves endothelial function, as well as increases ANP and NO secretion. The increase in blood glucose and epinephrine, which is caused by stress, affects NOS activity. The relief by labor analgesia can increase NO levels. Since average ET-1 concentration is lower than those of ANP and NO (unit: pg), ET-1-mediated ANP and NO increase will counteract the vasodilative effect of ET-1 through negative feedback. On the whole, ELA is helpful to improve placental circulation [25, 26]. In this study, the effects of ELA on umbilical artery blood NO, ANP, and ET-1 at different stages of labor were observed. The results showed that levels of the three were remarkably higher at the latent phase than those at the active phase. It is suggested that ELA from the latent phase is more helpful to increase NO, ANP, and ET-1 concentrations, which may be because from this phase, the onset time of analgesic drugs is longer, and the effect on placental blood vessels is more sustained. More beneficial to the improvement of placental microcirculation and the shortening of stages of labor, the improvement of the three will not affect the microcirculation and thus form adverse effects on delivery prognosis due to the longer onset time from this phase. The miRNA-146b level in the breast milk was remarkably higher, which was about 5.93 ± 0.48. The average VAS scores at the active phase and the second stage of labor were remarkably lower, which were 2.15 ± 0.22 and 2.37 ± 0.68, respectively.

The component of human milk has individual differences, possibly affected by the mother's age, regions, economy, nutrition, and modes of delivery. Expressed in various organs, tissues, and body fluids of human beings, miRNAs are involved in a series of important life processes such as the regulation of cell proliferation and differentiation, immune defense, and tumorigenesis [27]. MiR-146b, mainly through inhibiting the expression of toll-like receptors and intermediate molecules of nuclear factor-*κ*B pathway, inhibits the production of tumor necrosis factor-*α* and other proinflammatory cytokines [28] and thereby prevents the excessive immune and inflammatory responses of the body. Finally, we compared the miR-146b level in the breast milk between the two groups. The level was remarkably higher in the observation group (*P* < 0.05). However, we did not study the specific mechanism of this MiR, so it is hoped that in-depth analysis will be conducted in future studies.

In summary, ELA starting from latent phase can improve the miRNA-146b level in maternal breast milk, alleviate labor pain of parturients, and shorten stages of labor, so it is worthy of clinical promotion.

## Figures and Tables

**Figure 1:** Comparison of NO, ANP, and ET-1 levels.

**Figure 2:** Comparison of VAS scores at different time points.

**Table 1:** Comparison of general information (*n* (%))/(($\bar{x}$ ± sd).

Factors	Observation group (*n* = 65)	Control group (*n* = 54)	*t*/*χ*^2^ value	*P*
Age (years)	26.83 ± 3.81	27.49 ± 3.11	1.021	0.309
Gestational weeks (weeks)	36.62 ± 1.42	36.39 ± 1.66	0.815	0.417
BMI (kg/m^2^)	23.48 ± 0.46	23.42 ± 0.58	0.629	0.530
Types of parturients			0.449	0.503
Primiparas	51 (78.46)	45 (83.33)		
Multiparas	14 (21.54)	9 (16.67)		
Systolic blood pressure (mmHg)	153.86 ± 5.32	153.18 ± 4.85	0.722	0.472
Diastolic blood pressure (mmHg)	102.51 ± 4.27	101.76 ± 3.40	1.044	0.298

**Table 2:** Comparison of labor duration ($\bar{x}\pm \text{sd}$).

Groups	*n*	First stage of labor (min)		Second stage of labor (min)	Third stage of labor (min)
		Latent phase	Active phase		
Observation group	65	327.76 ± 83.89	75.80 ± 29.55	64.83 ± 15.52	7.83 ± 3.66
Control group	54	553.75 ± 88.81	83.98 ± 34.15	67.65 ± 18.67	7.17 ± 3.52
*t*	—	14.250	1.401	0.900	0.996
*P*	—	<0.001	0.164	0.370	0.321

**Table 3:** Comparison of modes of delivery (*n* (%)).

Groups	*n*	Eutocia	Cesarean section	Forceps delivery
Observation group	65	59 (90.77)	6 (9.23)	0 (0.00)
Control group	54	48 (88.89)	6 (11.11)	0 (0.00)
*χ* ^2^	—	0.115	0.115	—
*P*	—	0.735	0.735	—

**Table 4:** Comparison of NO, ANP, and ET-1 levels ($\bar{x}\pm \text{sd}$).

Groups	*n*	NO (*μ*mol/L)	ANP (ng/ml)	ET-1 (pg/ml)
Observation group	65	31.45 ± 4.42	346.87 ± 35.57	88.94 ± 12.96
Control group	54	27.43 ± 3.38	325.87 ± 32.76	78.25 ± 11.28
*t*	—	5.482	3.323	4.748
*P*	—	<0.001	0.001	<0.001

**Table 5:** Comparison of VAS scores at different time points ($\bar{x}\pm \text{sd}$).

Groups	*n*	First stage of labor (min)		Second stage of labor (min)	Third stage of labor (min)
		Latent phase	Active phase		
Observation group	65	2.52 ± 0.67	2.15 ± 0.22	2.37 ± 0.68	2.38 ± 0.51
Control group	54	2.69 ± 0.59	3.42 ± 0.58	3.58 ± 0.63	2.45 ± 0.88
*t*	—	1.454	16.310	9.990	0.541
*P*	—	0.149	<0.001	<0.001	0.589

**Table 6:** Comparison of adverse reactions (*n* (%)).

Groups	*n*	Respiratory depression	Nausea and vomiting	Numbness of limbs
Observation group	65	0 (0.00)	12 (18.46)	2 (3.08)
Control group	54	0 (0.00)	3 (5.56)	3 (5.56)
*χ* ^2^	—	—	4.460	0.450
*P*	—	—	0.035	0.502

**Table 7:** Comparison of miRNA-146b level.

Groups	*n*	MiR-146b
Observation group	65	5.93 ± 0.48
Control group	54	5.42 ± 0.52
*T*	—	5.556
*P*	—	<0.001

## Data Availability

The datasets used and/or analyzed during the current study are available from the corresponding author on reasonable request.
